# Two-Dimensional Ultrasound and Triplane Tissue Doppler Ultrasound of Patients with Severe Preeclampsia

**DOI:** 10.1155/2022/3384713

**Published:** 2022-06-20

**Authors:** Huili Tong, Yafeng Tian

**Affiliations:** Department of Obstetrics, Weinan Maternal and Child Health Care Hospital, Weinan, 714000 Shaanxi, China

## Abstract

This study was to investigate the cardiac function characteristics under two-dimensional ultrasound and triplane tissue Doppler imaging (TDI) of patients with severe preeclampsia (SPE). 28 SPE patients with singleton pregnancy from January 2018 to December 2020 were included in the SPE group. 25 healthy nonpregnant women of reproductive age were taken as the control group (Ctrl group), and 26 normal pregnant women with singleton pregnancy were selected as the normal group (Norm group); all the research objects underwent ultrasonography. The morphological and functional indexes of left and right ventricles were compared among the cases in different groups. The results showed that the left ventricular end-diastolic period diameter (LVEDd), left ventricular relative wall thickness (LV-RWT), left ventricular mass index (LVMi), left anterior descending (LAd), left ventricular *E*/*e* and *e*/*a* values, right ventricular diameter (RV-D), right ventricular anterior wall thickness (RVAW), *a* value, right atrial septum (RA-S), pulmonary artery systolic pressure (PASP), left ventricular end-systolic period diameter (LVEds), interventricular septal thickness (IVSd), posterior wall thickness (PWd), end-diastolic period volume (EVD), end-systolic period volume (ESV), relative wall thickness (RWT), sphericity index (SpI), left atrium volume index (LAVi), and *E*/*e* value of patients in the SPE group were higher than those in the Ctrl group and the Norm group (*P* < 0.05). The mitral annular plane systolic excursion (MAPSE), *s* value, tricuspid annual plane systolic excursion (TAPSE), ratio of early diastolic blood flow velocity to late diastolic blood flow velocity (*E*/*A*), ratio of peak early diastolic velocity to peak late diastolic velocity (*e*/*a*), peak early diastolic velocity (*e*), and ejection fraction (EF) of the SPE group were lower than those of the Ctrl group and the Norm group (*P* < 0.05). The ratio of mitral valve early diastolic blood flow velocity to peak early diastolic velocity (*E*/*e*) of the Norm group was higher than that of the Ctrl group (*P* < 0.05). In two-dimensional ultrasound of the SPE group, the maximum difference in time from the start to the peak of systole (Ts) of the right ventricle between the basal and middle segments of the lateral wall and that of interventricular septum (RV-Ts-max) was 31.56 ± 0.39%. The maximum difference in time to peak of early diastole (Te) under the same condition (RV-Te-max) was 47.16 ± 0.19%. Left ventricular LV-Ts-max and LV-Te-max were 9.83 ± 0.80% and 8.37 ± 0.68%, respectively, in triplane TDI, which were considerably higher than those in the Ctrl and Norm groups (*P* < 0.05). It suggested that two-dimensional ultrasound and triplane TDI could reflect the ventricular morphology as well as diastolic and systolic function injury in patients, which offered a reference basis for the diagnosis of SPE.

## 1. Introduction

Preeclampsia (PE) is a pregnancy-induced hypertension syndrome, which often involves multiple organs [1]. The incidence of PE is relatively high, as the global incidence reaches 3% to 8%, with about 12.5% of maternal deaths each year due to PE [2]. PE can cause increased peripheral blood resistance in pregnant women, decreased cardiac output (CO), and even heart failure, liver and kidney damage, brain damage, and death ultimately of pregnant women [3, 4]. PE is divided into mild and severe types according to the severity of the disease; in particular, severe preeclampsia (SPE) can bring about complications such as placental abruption and disseminated intravascular coagulation. SPE has the characteristics of complex pathogenetic condition, rapid development, and many complications, causing damage to systemic organs in different degrees and increasing the risk of vascular system damages [5].

At present, there is no uniform standard for the diagnosis and prediction of PE. In clinical practice, changes in high-risk factors, molecular markers, and biochemical indexes are often used for preliminarily prediction of PE. The current research outcomes suggest that the cardiac structure and function of SPE patients are significantly different from those of normal pregnant women [6]. Therefore, SPE can be diagnosed by evaluating cardiac function and its structural characteristics. With the development of imaging technology in recent years, echocardiography has been widely used in clinical diagnosis due to its noninvasiveness, low cost, low radiation, and simple operation. Traditional echocardiography has obvious errors in cardiac cycle assessment, so it is incapable to show the size of the cardiac chambers and to detect cardiac damage [7]. Two-dimensional Doppler echocardiography can overcome the shortcomings of traditional echocardiography and give cardiac function indexes, but it still has obvious limitations in the evaluation of the left ventricle (LV) [8]. Triplane tissue Doppler imaging (TDI) has fast imaging speed and high image resolution and overcomes the interference of respiratory motion [9]. Nowadays, triplane TDI has been widely used in the diagnosis of congenital heart diseases, pulmonary embolism, pulmonary hypertension, and other diseases [10].

In short, both two-dimensional ultrasound and triplane TDI have significant advantages in cardiac function assessment, but there are few studies conducted on the ultrasound characteristics of two-dimensional ultrasound and triplane TDI in the diagnosis of SPE. Singleton pregnancy SPE patients were selected as the research objects. Both healthy nonpregnant women and healthy pregnant women were invited as controls to analyze the two-dimensional ultrasound and triplane TDI characteristics of SPE patients, so as to provide a reference for the clinical diagnosis of SPE patients.

## 2. Materials and Methods

### 2.1. Research Objects

Convenience sampling was adopted to choose 28 singleton pregnancy SPE patients who were examined in the hospital from January 2018 to December 2020, and they were taken as the research objects (SPE group). They had an age range of 23-41 years old, with an average age of 30.17 ± 6.85 years old; the gestational age ranged from 21 to 37 weeks, and the average gestational age was 30.52 ± 0.69 weeks. Given the following diagnostic criteria for SPE [11], the patients were complicated with any of the conditions below in addition to hypertension and proteinuria after 20 weeks of gestation. (1) The serum creatinine ≥ 1.2 mg/dL. (2) Their proteinuria ≥ 2.0 g/24 hours, or the random protein ≥ (++). (3) Systolic blood pressure ≥ 160 mmHg and/or diastolic blood pressure ≥ 110 mmHg. (4) The platelet count < 100, 000/mL. (5) The patients had persistent headache or other brain or visual disturbances. (6) The patients were detected with elevated serum aminotransferase level. (7) They had the elevated lactate dehydrogenase. (8) They suffered from persistent epigastric pain. The patients' blood pressure returned to normal within 12 weeks postpartum, and they had no history of other heart disease and chronic diseases. Patients with cardiovascular and cerebrovascular diseases and other chronic diseases before pregnancy were excluded. The experimental process had been approved by the Ethics Committee of the hospital, and the objects included signed the informed consents.

25 healthy nonpregnant women of reproductive age, who came to our hospital for physical examination during the same period, were selected as the control group (Ctrl group). They had an age of 20-43 years old and an average age of 30.68 ± 5.49 years old. The inclusion criteria for women in the Ctrl group were as follows. They were healthy nonpregnant women with sinus rhythm, with no history of hypertension, coronary heart disease, and other cardiovascular diseases. They had no chronic diseases such as liver and kidney diseases.

Moreover, 26 normal pregnant women with singleton pregnancy, who came to the hospital for routine prenatal examination during the same period, were selected as the normal group (Norm group). Their age ranged between 20 and 43 years old, with the average age of 30.32 ± 4.92 years old; their gestational age was 21-37 weeks, and the average gestational age was 30.36 ± 0.78 weeks. Pregnant women with cardiovascular diseases, chronic liver and kidney disease history, and obstetric complications with fetal development were excluded.

### 2.2. Examination Methods of Two-Dimensional Echocardiography

All objects were in the left lateral decubitus position and were examined with color Doppler ultrasound diagnostic apparatus. In the breath-holding state, the two-dimensional M5S probe was used to collect ultrasound samples from the chordae tendineae level of the long-axis view of the parasternal LV, with the frequency of 1.7-3.4 MHz. Ultrasound images of three cardiac cycles were collected continuously and saved. Left ventricular end-diastolic period diameter (LVEDd), interventricular septal thickness (IVSd), left ventricular end-systolic period diameter (LVEds), and posterior wall thickness (PWd) were measured in echocardiographic mode. Mitral valve early diastolic blood flow velocity (*E*), mitral annular plane systolic excursion (MAPSE), mitral and tricuspid peak annular systolic velocity (*s*), tricuspid annual plane systolic excursion (TAPSE), peak early diastolic velocity (*e*), and peak late diastolic velocity (*a*) were also measured. Relative wall thickness (RWT) of LV and left ventricular mass index (LVMi) were then calculated [12]. All indexes were measured for three times, and the average values were taken.

### 2.3. Triplane TDI and Image Analysis

In the left lateral decubitus position, patients held their breath, a three-dimensional 4V-D probe was used to obtain the apical four-chamber view, and triplane TDI was performed. The images of three consecutive cardiac cycles were acquired. Left ventricular end-systolic volume (ESV), left ventricular end-diastolic volume (EDV), IVSd, end-diastolic left atrial volume (LAV), left ventricular ejection fraction (EF), left ventricular PWd at end diastole, left atrial volume index (LAVi), left ventricular CO, left ventricular spherical index (SpI), left ventricular mass (LVM), and *E* were measured. LVMi, RWT, and cardiac index (CI) were calculated [13].

### 2.4. Evaluation of Cardiac Motion Synchrony

Two-dimensional ultrasound was performed with the TDI curves. For each curve, the time from the start to the peak of systole (Ts) and the time to peak of early diastole (Te) were recorded. After heart rate normalization, the maximum difference in Ts and Te between the basal segment and the middle segment of lateral wall of the right ventricular (RV) and between the basal segment and the middle segment of the interventricular septum of RV (RV-Ts-max% and RV-Te-max%, respectively) were calculated. The curves of triplane quantitative tissue velocity imaging (QTVI) of the LV were automatically obtained through triplane TDI. The maximum difference of Ts and Te (LV-Ts-max% and LV-Te-max%) was also recorded.

### 2.5. Observation Index Detection

The general data such as age, gestational age, heart rate, systolic blood pressure, and diastolic blood pressure of women in the three groups were compared. The corresponding characteristics of the two-dimensional ultrasound and triplane TDI of the three groups were also analyzed. Finally, the differences in cardiac function-related indexes of the three groups were compared.

### 2.6. Statistical Methods

The experimental data was processed by SPSS 19.0 statistical software. The measurement data were expressed as the mean ± standard deviation ($\bar{x}\pm s$). The comparison of ultrasound-related indexes among the three groups was performed by one-way analysis of variance, and the pairwise comparison within the same group was performed by the least significant difference (LSD) method. The mean percentage of error was used to evaluate the repeatability, and *P* < 0.05 indicated that the difference was statistically significant.

## 3. Results

### 3.1. Comparison of General Data

As shown in Table 1, the general data such as age, height, body surface area (BSA), body mass index (BMI), gestational age, heart rate, systolic blood pressure, and diastolic blood pressure of the women in the SPE group, the Ctrl group, and the Norm group were compared. There were no significant differences in age, height, BSA, BMI, and gestational age among three groups (*P* > 0.05). The average heart rate of the Norm group was significantly higher than that of the Ctrl group (*P* < 0.05), while the average heart rate of the SPE group was lower than that of the Norm group (*P* < 0.05). There was also no significant difference in systolic and diastolic blood pressures between the Ctrl and Norm groups (*P* > 0.05). Both the systolic and diastolic blood pressures of the SPE group were higher than those of the Ctrl and Norm groups (*P* < 0.01).

### 3.2. Two-Dimensional Ultrasound Characteristics of SPE Patients

There was no abnormality in the size of the cardiac chambers and the inner diameter of the great vessels in patients with SPE. No abnormality was found in the thickness and range of motion of the ventricular septum as well as left ventricular walls. No abnormality was also found in the thickness, elasticity, and opening of each valve. Color flow showed no pathological regurgitation in each valve. The pulse Doppler sampling volume was under the mitral valve, and the diastolic bimodal laminar flow spectrum was recorded. The *E* peak (the filling peak of rapid filling of LV in the early diastole) was measured as 86 cm/s, the *A* peak (the filling peak of that in the late diastole) was 59 cm/s, and *E*/*A* > 1 (Figure 1).

### 3.3. Ultrasound Characteristics of Triplane TDI in Patients with SPE

In SPE patients, the anteroposterior diameter of the LV was 53 mm, while that of the left atrium was 38 mm. The size of the remaining cardiac chambers and the inner diameter of the great vessels were not abnormal. Besides, no abnormality was found in the thickness, elasticity, and opening range of valves. It was shown from color flow that there was no pathological regurgitation in any valve. The sampling volume of pulse Doppler was under the mitral valve, and the diastolic bimodal laminar flow spectrum was also recorded, with peak *E* of 78 cm/s, peak *A* of 108 cm/s, *E*/*A* < 1, and EF of 58% (Figure 2).

### 3.4. Comparison of Two-Dimensional Ultrasound Characteristics

The morphological and functional indexes of LV of the women in the SPE group, the Ctrl group, and the Norm group were compared and analyzed, as shown in Figure 3. The LVEDd and left anterior descending (LAd) of the SPE group were higher than those of the Ctrl group and the Norm group (*P* < 0.05). The MAPSE of the SPE group was lower than that of the Ctrl group and the Norm group (*P* < 0.05). The LV-RWT of women in the SPE group, the Ctrl group, and the Norm group were 0.41 ± 0.03 mm, 0.27 ± 0.01 mm, and 0.30 ± 0.02 mm, respectively. It was shown in Figure 3(a) that the LV-RWT of the SPE group was higher than that of the Ctrl group and the Norm group (*P* < 0.05). Higher LVMi was shown in the SPE group than in the Ctrl group and the Norm group (*P* < 0.05), and the LVMi in the Norm group was higher than that in the Ctrl group (*P* < 0.05). The value of *s* in the SPE group was lower than that in the Ctrl and Norm groups (*P* < 0.05), which could be observed in Figure 3(b). As shown in Figure 3(c), the values of *E*/*e* and *e*/*a* in the SPE group were also higher than those in the Ctrl group and the Norm group (*P* < 0.05), and the *E*/*e* value in the Norm group was higher than that in the Ctrl group (*P* < 0.05).

The morphological and functional indexes of the RV of women in the SPE group, the Ctrl group, and the Norm group were compared and analyzed, which were shown in Figure 4. The right ventricular diameter (RV-D) and right ventricular anterior wall thickness (RVAW) of the SPE group were higher than those of the Ctrl group and the Norm group (*P* < 0.05). The TAPSE values of women in the SPE, Ctrl, and Norm groups were 14.98 ± 1.22 mm, 18.05 ± 1.47 mm, and 18.82 ± 1.54 mm, respectively. TAPSE of the SPE group was lower than that of the Ctrl and Norm groups (*P* < 0.05). As shown in Figure 4(a), there was no significant difference in RV-D, RVAW, and TAPSE between the Ctrl group and the Norm group (*P* > 0.05). There was also no significant difference in the ratio of *s* value and *e* value among the SPE group, the Ctrl group, and the Norm group (*P* > 0.05). The *a* value of the SPE group was higher than that of the Ctrl group and the Norm group (*P* < 0.05), but no statistical difference in *a* value was found between the Ctrl group and the Norm group (*P* > 0.05), as it could be observed in Figure 4(b). The values of *E*/*A* and *e*/*a* in the SPE group were lower than those in the Ctrl group and the Norm group (*P* < 0.05), but those in the Ctrl group were not significantly different from those in the Norm group (*P* > 0.05), which was displayed in Figure 4(c). The right atrial septum (RA-S) value and pulmonary artery systolic pressure (PASP) of the SPE group were higher than those of the other two groups (*P* < 0.05), and no significant difference was shown in the RA-S and PASP between the Ctrl and Norm groups (*P* > 0.05), which were represented in Figures 4(d) and 4(e).

### 3.5. Comparison of Triplane TDI Characteristics

As shown in Figure 5, the left ventricular morphological indexes of women in the SPE group, the Ctrl group, and the Norm group were compared and analyzed. The LVEDd, LVEDs, and IVSd of the SPE group were higher than those of the Ctrl group and the Norm group (*P* < 0.05); but there was no significant difference in the three indexes between the Ctrl group and the Norm group (*P* > 0.05). PWd of women in the SPE, Ctrl, and Norm groups were 9.54 ± 0.78 mm, 6.48 ± 0.53 mm, and 6.35 ± 0.52 mm, respectively, from which the PWd of the SPE group was higher than that of the Ctrl group and the Norm group (*P* < 0.05). There is no statistical difference in PWd between the Ctrl and Norm groups (*P* > 0.05), as it could be found in Figure 5(a). In Figure 5(b), the end-diastolic period volume (EVD) and end-systolic period volume (ESV) in the SPE group were higher than those in the other two groups (*P* < 0.05), but there was no significant difference in EVD and ESV between the Ctrl group and the Norm group (*P* > 0.05). In Figure 5(c), the RWT and SpI of the SPE group were higher than those of the Ctrl and Norm groups (*P* < 0.05), and no significant difference was between the Ctrl group and the Norm group (*P* > 0.05). LVMi of women in the SPE, Ctrl, and Norm groups were 84.02 ± 6.86 g/m^2^, 60.27 ± 4.92 g/m^2^, and 69.84 ± 5.70 g/m^2^, respectively. As shown in Figure 5(d), the LVMi of the SPE group was higher than that of the other two groups (*P* < 0.05), and that of the Ctrl group and the Norm group was not significantly different (*P* > 0.05).

In Figure 6, the three-dimensional ultrasound left ventricular function indexes of women in the three groups were compared and analyzed. It was shown in Figure 6(a) that the *s* value and *e* value of the SPE group were lower than those of the Ctrl group and the Norm group (*P* < 0.05). The *a* value in the SPE group was higher than that in the Ctrl group and the Norm group (*P* < 0.05). There was no statistical difference in the *s* value, *e* value, and *a* value between the Ctrl group and the Norm group (*P* > 0.05). LAVi and *E*/*e* value of the SPE group were higher than those of the other two groups (*P* < 0.05), while those of the women in the Ctrl group and the Norm group were not significantly different (*P* > 0.05), which were displayed in Figures 6(b) and 6(c). From Figure 6(d), EF of the SPE group was significantly lower than that of the Ctrl group and the Norm group (*P* < 0.05), and no significant difference in EF was discovered between the Ctrl group and the Norm group (*P* > 0.05). The CI value of women in the SPE group, the Ctrl group, and the Norm group was 2.48 ± 0.20 L/min/m^2^, 2.38 ± 0.19 L/min/m^2^, and 2.45 ± 0.20 L/min/m^2^, respectively. As shown in Figure 6(e), there was no significant difference in the CI values between the SPE, Ctrl, and Norm groups (*P* > 0.05).

### 3.6. Analysis of Left and Right Ventricular Motion Synchrony

The synchrony of the LV and RV of the women in the three groups was compared and analyzed in Figure 7. The two-dimensional ultrasound RV-Ts-max and RV-Te-max of the SPE group were 31.56 ± 0.39% and 47.16 ± 0.19%, respectively, which were significantly higher than those of the Ctrl group and the Norm group (*P* < 0.05). There was no statistical difference in RV-Ts-max and RV-Te-max between the Ctrl group and the Norm group (*P* > 0.05), as shown in Figure 7(a). The LV-Ts-max and LV-Te-max in the SPE group were 9.83 ± 0.80% and 8.37 ± 0.68%, respectively, significantly higher than those in the other two groups (*P* < 0.05); but those of the Ctrl group were not statistically different from those of the Norm group (*P* > 0.05), which is represented as Figure 7(b).

## 4. Discussion

PE refers to a hypertensive syndrome that occurs after 20 weeks of gestation, which returns to normal levels by 12 weeks postpartum generally [14]. Imaging methods currently used in the assessment of cardiac morphology and function in pregnant women include left ventriculography, radionuclide cardiac blood pool imaging, cardiac magnetic resonance imaging, and ultrasonography [15]. Left ventriculography is the current gold standard for evaluating cardiac function, but it is an invasive operation [16]. Ultrasonography is widely used in clinical diagnosis due to its noninvasiveness, low radiation, and simple operation [17]. The clinical symptoms of SPE are more severe, so the impact on the cardiovascular system is more significant [18]. Two-dimensional ultrasound and triplane TDI ultrasound were used to analyze the clinical characteristics of SPE patients and the changes in morphology and function indexes of LV and RV. The results showed that LVEDd, LV-RWT, LVMi, LAd, left ventricular *E*/*e* value, left ventricular *e*/*a* value, RV-D, RVAW, *a* value, RA-S, and PASP of the SPE group were higher than those of the Ctrl group and the Norm group (*P* < 0.05). The MAPSE, *s*, TAPSE, *E*/*A*, and *e*/*a* value of the SPE group were lower than those of the other two groups (*P* < 0.05). The *E*/*e* value of the Norm group was higher than that of the Ctrl group (*P* < 0.05). These results suggested that the left ventricular systolic function of women during normal pregnancy had no significant change compared with nonpregnant women of reproductive age, which was different from the results of Shahid et al. [19]. The gestational age of the included pregnant women was relatively small, and the left ventricular systolic function was in a compensated phase, so there was no significant difference compared with nonpregnant women of reproductive age. Furthermore, it could be found that the *E*/*e* value of women during normal pregnancy was higher than that of the Ctrl group, indicating that diastolic function decreased during pregnancy. The *e*/*a* value of SPE patients was significantly lower, which perhaps because of the increase of LVMi and afterload of LV, so that a compensatory response occurred in the left atrium with increased systole [20]. There was no statistical difference in the morphological and functional indexes of the RV between the Ctrl group and the Norm group. This was because the blood volume of the pregnant women in the Norm group increased, but the vascular resistance of the pulmonary vascular bed decreased, so the RV morphological and functional indexes had no significant change. Sarno et al. [21] pointed out that when the blood volume of LV and RV increased, the pressure of LV increased significantly, but the pressure of RV did not change obviously. This was because the RV had a stronger receptivity than the LV. However, the two-dimensional ultrasound here was mainly used to research the RV, so there was no significant change in the related indexes of the Ctrl group and the Norm group.

With the comparison of the morphological and functional indexes of left ventricular three-dimensional ultrasound of women in different groups, it was found that the LVEDd, LVEDs, IVSd, PWd, EVD, ESV, RWT, SpI, LVMi, *a* value, LAVi and *E*/*e* value of the SPE group were all higher than those of both the Ctrl group and the Norm group (*P* < 0.05), while the *s*, *e*, and EF values of the SPE group were lower than those of the other two groups (*P* < 0.05). In SPE patients, the ventricular wall was thickened, the LVMi and SpI increased, and the ventricular cavity was enlarged. Thus, it was speculated that the LV of SPE patients might suffer from centrifugal hypertrophy, which was different from the results obtained by Adekanmi et al. [22] and Sarno et al. [23]. The reason might be the varied severity of the disease of the SPE patients. The *E*/*e* value is a good measure of left ventricular diastolic function, and left atrial remodeling is significantly correlated with left ventricular diastolic function [24]. The ventricular ejection capacity was obstructed after hypervolemia in SPE patients, resulting in increased left ventricular filling pressure [25].

## 5. Conclusion

The analysis was performed of the cardiac function characteristics of two-dimensional ultrasound and triplane TDI ultrasound in patients with SPE. It was found from the results that SPE patients had right ventricular enlargement, ventricular wall hypertrophy, impaired cardiac diastolic and systolic function, and decreased left and right ventricular synchrony. However, there were still some shortcomings. For the grouping, no further analysis was made according to different gestational weeks, and no early-onset and late-onset typing studies were conducted on SPE patients. These factors would be researched one by one in the future stage. In conclusion, two-dimensional ultrasound and triplane TDI ultrasound could display the ventricular morphology, diastolic function injury, and systolic function injury in patients. Thus, a reference for the diagnosis of SPE could be provided as a consequence.

## Figures and Tables

**Figure 1:** Two-dimensional ultrasound characteristics of patients with SPE (gestational age of 26 weeks).

**Figure 2:** Triplane TDI ultrasound characteristics of patients with SPE (gestational age of 26 weeks).

**Figure 3:** Comparison of left ventricular indexes in morphology and function by two-dimensional ultrasound in different groups. (a) Comparison of LVEDd, LAd, MAPSE, and LV-RWT in different groups by two-dimensional ultrasound. (b) Comparison of LVMi and *s* in different groups by two-dimensional ultrasound. (c) Comparison between *E*/*e* and *e*/*a* of LV by two-dimensional ultrasound in different groups. ^∗^Compared with the Ctrl group, *P* < 0.05; ^#^compared with the Norm group, *P* < 0.05.

**Figure 4:** Comparison of morphological and functional indexes of the RV under two-dimensional ultrasound in different groups: (a) comparison of RV-D, RVAW, and TAPSE; (b) comparison of *s*, *e*, and *a* value; (c) *E*/*A* ratio compared with *e*/*a* value; (d) comparison of RA-S; (e) comparison of PASP. ^∗^Compared with the Ctrl group, *P* < 0.05; ^#^compared with the Norm group, *P* < 0.05.

**Figure 5:** Comparison of left ventricular morphological indexes of triplane TDI in different groups. (a) Comparison of LVEDd, LVEDs, IVSd, and PWd. (b) Comparison of EVD and ESV. (c) Comparison of RWT and SpI. (d) Comparison of LVMi. ^∗^Compared with the Ctrl group, *P* < 0.05; ^#^compared with the Norm group, *P* < 0.05.

**Figure 6:** Comparison of left ventricular function indexes under triplane TDI in different groups. (a) Comparison of *s*, *e*, and *a* values in different groups. (b) Comparison of LAVi in different groups. (c) Comparison of *E*/*e*. (d) Comparison of EF in different groups. (e) Comparison of CI values in different groups. ^∗^Compared with the Ctrl group, *P* < 0.05; ^#^compared with the Norm group, *P* < 0.05.

**Figure 7:** Comparison of left and right ventricular motion synchrony. (a) Comparison of RV-Ts-max and RV-Te-max of the RV under two-dimensional ultrasound in different groups. (b) Comparison of LV-Ts-max and LV-Te-max of LV under triplane TDI ultrasound in different groups. ^∗^Compared with the Ctrl group, *P* < 0.05; ^#^compared with the Norm group, *P* < 0.05.

**Table 1:** Comparison of clinical data of women in different groups ($\bar{x}\pm s$).

Items	SPE group (*n* = 28)	Ctrl group (*n* = 25)	Norm group (*n* = 26)
Age (years old)	30.17 ± 6.85	30.68 ± 5.49	30.32 ± 4.92
Height (cm)	162.82 ± 2.97	163.04 ± 3.32	162.25 ± 3.26
BSA (m^2^)	1.75 ± 0.31	1.81 ± 0.24	1.78 ± 0.19
BMI (kg/m^2^)	22.34 ± 2.12	22.86 ± 3.19	23.05 ± 2.63
Gestational age (weeks)	30.52 ± 0.69	/	30.36 ± 0.78
Heart rate (beats/min)	79.08 ± 7.85^#^	74.76 ± 7.65	86.87 ± 8.52^∗^
Systolic blood pressure (mmHg)	143.52 ± 15.26^#^^∗^	106.95 ± 9.82	105.03 ± 10.03
Diastolic blood pressure (mmHg)	98.18 ± 9.82^#^^∗^	71.64 ± 7.74	72.01 ± 8.61

^∗^Compared with the Ctrl group, *P* < 0.05; ^#^compared with the Norm group, *P* < 0.05.

## Data Availability

The data used to support the findings of this study are available from the corresponding author upon request.
